This article has been retracted.

# Gene expression analysis indicates CB1 receptor upregulation in the hippocampus and neurotoxic effects in the frontal cortex 3 weeks after single-dose MDMA administration in Dark Agouti rats

**DOI:** 10.1186/1471-2164-14-930

**Published:** 2013-12-30

**Authors:** Peter Petschner, Viola Tamasi, Csaba Adori, Eszter Kirilly, Romeo D Ando, Laszlo Tothfalusi, Gyorgy Bagdy

**Affiliations:** 1 Department of Pharmacodynamics, Semmelweis University, H-1089 Nagyvarad ter 4., Budapest, Hungary; 2 Department of Genetics, Cell- and Immunobiology, Semmelweis University, H-1089 Nagyvarad ter 4., Budapest, Hungary; 3 MTA-SE Neuropsychopharmacology and Neurochemistry Research Group, Budapest, Hungary

**Keywords:** MDMA, Ecstasy, Endocannabinoid, CB1, Addiction, Cognition, Memory, Rat, Gene expression, Microarray

## Abstract

**Background:**

3,4-methylenedioxymethamphetamine (MDMA, "ecstasy") is a widely used recreational drug known to impair cognitive functions on the long-run. Both hippocampal and frontal cortical regions have well established roles in behavior, memory formation and other cognitive tasks and damage of these regions is associated with altered behavior and cognitive functions, impairments frequently described in heavy MDMA users. The aim of this study was to examine the hippocampus, frontal cortex and dorsal raphe of Dark Agouti rats with gene expression arrays (Illumina RatRef bead arrays) looking for possible mechanisms and new candidates contributing to the effects of a single dose of MDMA (15 mg/kg) 3 weeks earlier.

**Results:**

The number of differentially expressed genes in the hippocampus, frontal cortex and the dorsal raphe were 481, 155, and 15, respectively. Gene set enrichment analysis of the microarray data revealed reduced expression of 'memory’ and 'cognition’, 'dendrite development’ and 'regulation of synaptic plasticity’ gene sets in the hippocampus, parallel to the upregulation of the CB1 cannabinoid- and *Epha4*, *Epha5*, *Epha6* ephrin receptors. Downregulated gene sets in the frontal cortex were related to protein synthesis, chromatin organization, transmembrane transport processes, while 'dendrite development’, 'regulation of synaptic plasticity’ and 'positive regulation of synapse assembly’ gene sets were upregulated. Changes in the dorsal raphe region were mild and in most cases not significant.

**Conclusion:**

The present data raise the possibility of new synapse formation/synaptic reorganization in the frontal cortex three weeks after a single neurotoxic dose of MDMA. In contrast, a prolonged depression of new neurite formation in the hippocampus is suggested by the data, which underlines the particular vulnerability of this brain region after the drug treatment. Finally, our results also suggest the substantial contribution of CB1 receptor and endocannabinoid mediated pathways in the hippocampal impairments. Taken together the present study provides evidence for the participation of new molecular candidates in the long-term effects of MDMA.

## Background

Ecstasy (3,4-methylenedioxymethamphetamine, MDMA) is an amphetamine derivative widely abused for its euphoric and entactogenic effects in developed countries [1,2]. The acute indirect monoaminergic agonist effects of MDMA are mainly mediated by an increase in serotonergic, noradrenergic and dopaminergic neurotransmission of the brain by reversing transmembrane transporter functions, which are normally responsible for the uptake of neurotransmitters from the synaptic cleft [1-4]. However, in the long-run, a decrease in serotonergic markers was reported in experimental animals and also in human users suggesting a long-term selective vulnerability of the serotonergic system [2,5-7]. Functional deficits could also be observed in humans and in rodents, e.g. impaired decision making, sleep disturbances, increased anxiety and impulsivity levels, elevated aggression, learning and memory impairments and depression [2,6,8-10]. Additionally to the selective damage observed in serotonergic neurons, MDMA may also cause more wide-spread neurotoxicity, possibly by its hyperthermic effect and the production of toxic metabolites and free radicals or via the disruption of local cerebral blood flow and glucose utilization, which might cause alterations in the nutrition-supply of neurons [5,11-19].

The serotonergic projections in the mammalian brain, the primary targets of MDMA’s effects in rats, originate from the raphe nuclei in the brainstem. Dorsal (DR) and medial raphe nuclei innervate upper brain structures, including the frontal cortical regions and the hippocampus (HC) [20-23]. The frontal cortex (FC) plays major roles in risk evaluation [24], executive functioning [24,25], and working memory [26-28], while its malfunctions may be associated with neuropsychiatric diseases [24,29]. At the same time, HC has a pivotal role in contextual and hereby spatial memory formation [23,30] thus all of the latter regions are candidates for long-run functional deficits caused by MDMA.

Parallel to the neuronal damage, however, neuroprotective mechanisms also occur and, later in time, recovery processes also may begin. Heat-shock proteins (HSPs) can ameliorate the damage caused by cellular stress of different origin, e.g. hyperthermia, ischemia, or excessive production of free radicals [31]. Elevated levels of HSP 27 in the FC and HC 3 days after MDMA treatment was demonstrated by Adori et al. and this elevation persisted until at least 7 days in the HC but normalized in the FC by this time [5]. Brain-derived neurotrophic factor (BDNF), a well-characterized member of neurotrophic factors, is involved in several processes maintaining central nervous system (CNS) functions like dendritic arborization, synaptogenesis and activity-dependent potentiation (for reviews see [32] and [33]). A study elucidating MDMA’s effects on BDNF mRNA expression reported ever increasing elevations in FC up to 7 days after MDMA administration while in the HC a decrease was evident [34]. Investigation of MDMA’s long-term effects revealed that in the parietal cortex BDNF protein levels peaked at 8 weeks after an initial decline but in the HC no significant change could be reported [35]. All of the latter results suggest different recovery capacities of the HC and FC, but the detailed biochemical mechanisms responsible for these differences remained so far less investigated at later time points. We speculated that these consequences might be already visible at 21 days following a single dose of MDMA thus we performed our analysis 3 weeks after drug administration to investigate both the recovery processes and the downstream mediators of damages.

Studies examining transcriptional changes following MDMA administration are scarce, only few reports evaluated alterations in mRNA levels of genes which were assumed to be related to MDMA effects [6,10,35-41].

Thus, the aim of this study was to address the downstream transcriptional consequences of MDMA’s effects and to find possible new targets of regulatory mechanisms by using large-scale gene expression profiling in the HC, FC, and DR regions of DA rats 21 days after a single-dose MDMA administration. Additionally, we also addressed whether signs of functional recovery on the molecular level can occur in the FC and HC regions and if so, whether they differ in quality or quantity in these two regions. Furthermore, for comparable results with our earlier studies, we used the same dosage regimen (15 mg/kg) in the Dark Agouti (DA) rat strain, which represents the human "poor metabolizer" phenotype [42].

## Results

### General overview of gene expression alterations

Comparison of the gene expression profiles showed 615 differentially expressed genes in the MDMA treated group compared to the saline control (minimum probability of positive log ratio [MinPplr] < 0.001) (Figure 1). In the HC region 481 genes showed altered expression, 310 and 171 genes were up- or downregulated, respectively. From 155 significant genes in the FC region 89 were up- and 66 downregulated. Only 14 unique genes were altered in the DR region, 3 showed elevated expression and the remaining 11 showed a decrease compared to the control group. All genes emphasized below were selected by individual considerations of MDMA’s known effects and related literature data. For full results see Additional file 1: Table S1.

**Figure 1:** **Venn-diagram representation of significantly altered mRNAs.** Venn-diagrams showing the number of significantly (minimum probability of positive log ratio (MinPplr) < 0.001) up- or downregulated genes in the hippocampus (HC), frontal cortex (FC) and dorsal Raphe (DR) of Dark Agouti (DA) rats 3 weeks after a single-dose of 3,4-methylenedioxymethamphetamine (MDMA) (15 mg/kg, intraperitoneally). Altogether 615 genes’ showed altered expression, 481, 155, 14 genes in the HC, FC, DR regions, respectively. Among them only 1 genes’ expression altered significantly in all three regions and 36 genes differed significantly compared to saline controls in both the FC and HC groups. See text for further details.

The GSEA analysis revealed 18, 55 and 1 differentially regulated gene sets in the HC, FC and DR regions, respectively.

### Hippocampus

#### Differentially expressed genes

Changes in major hippocampal neurosignaling pathways included an elevation in the type 1 cannabinoid receptor (*Cnr1,* CB1), glutamatergic AMPA3 (*Ampa3*) and GRIN2A receptor mRNA levels (*Gria3*), parallel with an increased expression of *Epha4* (*LOC316539)*, *Epha5* and *Epha6* receptors, members of ephrin signaling. Additionally the GABA-A receptor subunit (*Gabre*) was downregulated. A variety of calcium signaling pathway members were dysregulated, the type 2 inhibitor of the calcium/calmodulin dependent protein kinase II (C*amk2n2*) was downregulated, while *Camk2n1* and calcium/calmodulin dependent kinase genes showed upregulations (*Camk2g*, *Camk2b*). In accordance, the mRNA levels of *Atp2b3*, *Atp2b1* calcium transporting ATP-ases and *Slc5a3*, an inositol transporter was also increased. Some of the voltage-gated potassium transporter genes (*Kcnd2*, *Kcnc2*) were upregulated (see Additional file 1: Table S1 for full results).

#### Gene set enrichment analysis

The GSEA analysis revealed altogether 18 differentially represented gene sets in the HC region, including both the Msig DB C5 gene set database and individually chosen gene sets according to the literature (Additional file 2: Table S2), thus, protein kinase activity (GO:0004672), protein kinase binding (GO:0019901), protein amino acid phosphorylation (GO:0006468), symporter activity (GO:0015293), phosphorylation (GO:0016310), secondary active transmembrane transporter activity (GO:0015291), dendrite development (GO:0016358), memory (GO:0007613), regulation of synaptic plasticity (GO:0048167), cellular response to retinoic acid (GO:0071300), positive regulation of neuron projection development (GO:0010976), regulation of synaptic transmission, glutamatergic (GO:0051966), regulation of long-term neuronal synaptic plasticity (GO:0048169), positive regulation of neuron differentiation (GO:0045666), neuron projection terminus (GO:0044306), regulation of excitatory postsynaptic membrane potential (GO:0060079), cognition (GO:0050890) and synaptosome (GO:0019717) gene sets were downregulated (see Additional file 3: Table S3 for detailed results). We also used *in silico* GSEA network analysis (Figure 2) on significantly enriched gene ontology (GO) terms, which represents functional connectivity and was applied to determine biologically relevant processes shown in Table 1. From the 18 differentially expressed gene sets 'memory’ and 'cognition’ and multiple pathways related to the molecular function of kinases has to be emphasized among processes related to synaptic plasticity and dendrite and synapse development. The regulation of glutamatergic neurotransmission was also downregulated (Table 1, in all cases, p < 0.05, and false discovery rate (FDR) < 0.25). Figure 3 summarizes some of the main findings of the GSEA analysis.

**Figure 2:** **Network analysis of the GSEA results in the Hippocampus.** The network shows significantly (nominal p < 0.05, false discovery rate < 0.25) enriched gene ontology (GO) terms in the gene set enrichment (GSEA) analysis in the hippocampus (HC) of Dark Agouti rats 3 weeks after a single-dose (15 mg/kg, intraperitoneal) 3,4-methylenedioxymethamphetamine (MDMA) administration. Blue circles represent the downregulation of the associated terms, while red circles would represent upregulations. The size of the nodes is proportional with the number of genes in the GO term and the thickness of the edges between lines represents the similarity coefficient. All processes in the HC are downregulated, and two well characterized groups of processes emerge. On one hand the processes related to cognition and memory, e.g. regulation of synaptic plasticity, dendrite development and regulation of glutamatergic synaptic transmission gene sets form diverse groups. On the other hand the processes related to kinase activity form another network. See text for further details.

**Table 1:** Biologically relevant processes with enriched gene sets in the hippocampal region

**Biological process**	**Number of enriched gene sets related to the term**	**Direction**
Protein phosphorilation	4	⬇
Dendrite and synapse development	4	⬇
Synaptic plasticity	4	⬇
Transmembrane transport	2	⬇
Others	2	⬇
Memory, cognition	2	⬇

This table summarizes the biological processes significantly altered in the hippocampus of Dark Agouti rats after a single-dose 3,4-methylenedioxymethamphetamine (MDMA) treatment (15 mg/kg, intraperitoneal) 3 weeks earlier. The processes were created based on the network analysis of gene set enrichment (GSEA) analysis and individual considerations. All significantly enriched GO terms are included in one of the processes. Downward arrows represent downregulations. See text for further details.

**Figure 3:** **A schematic representation of MDMA’s sites of action in the Hippocampus.** This figure summarizes the effects of a single-dose (15 mg/kg, intraperitoneal) of 3,4-methylenedioxymethamphetamine (MDMA) 3 weeks earlier on hippocampal neurons in Dark Agouti rats. Three distinct processes were identified marked by text boxes on the figure, phosphorylation- and dendrite development-related gene sets and gene sets involved in the proper synaptic functioning were downregulated (signed with red crosses at possible sites of action). These processes can be bound to memory and cognition gene sets (downregulated alike) through a single mediator, namely the type 1 cannabinoid receptor (CB1). Accordingly, single-dose MDMA administration 3 weeks earlier resulted in elevated CB1 mRNA levels in the hippocampus. It has to be noted that compared to the frontal cortical region (Figure 5), where rather intracellular signaling mechanisms were influenced, in the HC gene sets related to the connectivity of neurons were damaged. See text for further details.

### Frontal cortex

#### Differentially expressed genes

MDMA caused a significant underexpression of genes related to the calcium signaling pathways (*Camk2g* and *Camk1g*) and the ionotropic glutamate receptor, NMDA2B (*Grin2b*). The alpha subunit of the heat shock protein 1 (*Hspca*) and the heat shock factor 2 (*Hsf2*) were upregulated, similarly to the high-affinity glial glutamate transporter (*Slc1a3*) (see Additional file 1: Table S1 for full results).

#### Gene set enrichment analysis

Altogether 55 gene sets were differentially enriched after the single-dose MDMA treatment, containing both our literature-based, individually chosen (Additional file 2: Table S2) and Msig DB C5 gene sets. Additionally as in the case of HC, we also used GSEA network analysis on significantly enriched GO terms (Figure 4) to determine biologically relevant processes shown in Table 2. The upregulated gene sets included the response to hyperoxia (GO:0055093), positive regulation of synapse assembly (GO:0051965), regulation of synaptic plasticity (GO:0048167), growth factor activity (GO:0008083) and dendrite development (GO:0016358) gene sets. While organic acid transport (GO:0015849), carboxylic acid transport (GO:0046942), translation (GO:0006412), macromolecule biosynthetic process (GO:0009059), pattern specification process (GO:0007389), RNA binding (GO:0003723), hydro lyase activity (GO:0016836), intracellular protein transport (GO:0006886), establishment and or maintenance of chromatin architecture (GO:0006325), nuclear import (GO:0051170), protein import into nucleus (GO:0006606), intracellular transport (GO:0046907), cellular biosynthetic process (GO:0044249), structural molecule activity (GO:0005198), protein import (GO:0017038), amine transport (GO:0015837), isomerase activity (GO:0016853), amino acid transport (GO:0006865), biosynthetic process (GO:0009058), structural constituent of ribosome (GO:0003735), macromolecule localization (GO:0033036), protein localization (GO:0008104), nuclear membrane part (GO:0044453), protein transport (GO:0015031), nuclear transport (GO:0051169), nucleocytoplasmic transport (GO:0006913), establishment of protein localization (GO:0045184), protein targeting (GO:0006605), amino acid transmembrane transporter activity (GO:0015171), cell cycle arrest (GO:0007050), chromatin modification (GO:0016568), hematopoietin interferon class d200 domain cytokine receptor activity (GO:0004896), electron transport (GO:0006118), organic acid transmembrane transporter activity (GO:0005342), endopeptidase activity (GO:0004175), oxidoreductase activity (GO:0016491), ribonucleoprotein complex (GO:0030529), cysteine type peptidase activity (GO:0008234), negative regulation of growth (GO:0045926), protein processing (GO:0016485), carboxylic acid transmembrane transporter activity (GO:0046943), chromosome organization and biogenesis (GO:0051276), lipid transport (GO:0006869), cell cycle process (GO:0022402), nuclear part (GO:0044428), mitotic cell cycle (GO:0000278), protein-RNA complex assembly (GO:0022618), RNA processing (GO:0006396), nuclear envelope-endoplasmic reticulum network (GO:0042175), establishment of cellular localization (GO:0051649) gene sets were downregulated (see Additional file 3: Table S3 for detailed results). Classifying these gene sets into biological processes, the most prominent alterations were related to protein synthesis and protein localization within the neurons and contained 21 significantly dysregulated GO pathways, while 10 significantly enriched gene sets were involved in transport processes. All of these 31 gene sets, without exception, were downregulated in the FC region, together with gene sets responsible for chromatin maintenance. Among the upregulated gene sets in the FC, dendrite and synapse development and growth factor activity has to be emphasized 3 weeks after MDMA administration (Table 2, in all cases, p < 0.05, and FDR < 0.25). Figure 5 summarizes the main findings of the GSEA analysis.

**Figure 4:** **Network analysis of the GSEA results in the frontal cortex.** The network shows significantly (nominal p < 0.05, false discovery rate < 0.25) enriched gene ontology (GO) terms in the gene set enrichment (GSEA) analysis in the frontal cortex (FC) of Dark Agouti rats 3 weeks after a single-dose (15 mg/kg, intraperitoneal) 3,4-methylenedioxymethamphetamine (MDMA) administration. Blue and red circles represent down- and upregulation of the associated GO terms, respectively. The size of the nodes is proportional with the number of genes in the GO term and the thickness of the grey edges represents the number of common genes between two GO terms, if any. Most of the processes in the FC were downregulated. The cellular biosynthetic process and establishment of cellular localization GO terms are in central positions of two different groups while chromosome and chromatin organization, and transmembrane transport processes form the third and fourth group of tightly related, downregulated gene sets. These alterations suggest a general neurotoxic effect while the upregulation of gene sets related to synapse formation raises the possibility of a parallel running recovery process. The expression of the only immunologically related GO term was attenuated. See text for further details.

**Table 2:** Biologically relevant processes with enriched gene sets in the frontal cortical region

**Biological process**	**Number of enriched gene sets related to the process**	**Direction**
Protein synthesis and localization	21	⬇
Transmembrane transport	10	⬇
Nucleocytoplasmic transport	7	⬇
Cell growth	6	⬆⬇
Others	4	⬆⬇
Chromatine maintenance	3	⬇
Dendrite and synapse development	3	⬆
Oxidoreductase acitivity	2	⬇

This table summarizes the biological processes significantly altered in the frontal cortex (FC) of Dark Agouti (DA) rats after a single-dose 3,4-methylenedioxymethamphetamine (MDMA) treatment (15 mg/kg, intraperitoneal) 3 weeks earlier. The processes were created based on the network analysis of gene set enrichment (GSEA) analysis and individual considerations. All significantly enriched GO terms are included in one of the processes. Downward arrows represent down-, upward arrows represent upregulations. In some of the biological processes both up- and downregulated gene sets were present (mixed up- and downward arrows). See text for further details.

**Figure 5:** **A schematic representation of MDMA’s sites of action in the frontal cortex.** This figure summarizes the effects of a single-dose (15 mg/kg, intraperitoneal) 3,4-methylenedioxymethamphetamine (MDMA) administration 3 weeks earlier on the frontal cortex (FC) neurons of Dark Agouti rats. The text boxes mark the selected, grouped processes while red crosses represent the possible sites of action. Almost all of the genes involved in different levels of protein synthesis were downregulated, including nucleocytoplasmic transport, ribosome functioning, protein folding and localization and members in the transport of amino acids and lipids, basic constituents of the cells. These changes strongly suggest a wide-scale impairment of the cellular machinery. However, the formation of new neuronal connections can compensate for these effects (not depicted) on a different scale. See text for further details.

### Dorsal raphe

#### Differentially expressed genes

In the DR region the glycine neurotransmitter transporter (*Slc6a5*), the D-amino acid oxydase (*Dao1*) and the 11-beta-hydroxisteroid dehydrogenase (*Hsd11b1*) genes were downregulated among others (see Additional file 1: Table S1 for full results).

#### Gene set enrichment analysis

In the DR region only one gene set, namely caspase activation was significantly downregulated after the single-dose MDMA treatment. No upregulated gene sets could be observed (in all cases p < 0.05, and FDR < 0.25). The full results of the GSEA analysis in the DR region are shown in Additional file 3: Table S3.

### Heatmap analysis

The heatmap (Figure 6) shows genes after two-way hierarchical clustering comparing their expression levels among all three regions. It provides a different insight into the transcriptional changes after MDMA treatment. In the HC region nearly all of the genes were downregulated. In contrast, most of those genes that were downregulated in the FC were found to be upregulated in the HC, suggesting marked differences between the two regions. Changes in the DR were scant independently of alterations in the other two regions.

**Figure 6:** **Correlation between the microarray and the Fluidigm GEx PCR array data.** The figure summarizes the correlation between the logarithmic microarray data and the validation results for both the 200 ng and 500 ng samples. For validation purposes we used the polymerase chain reaction-based (PCR-based) Fluidigm GEx array with 19 genes and upon receiving the results, the numerical analysis was performed with the inbuilt corr.test function of the R statistical computing program. The results are in agreement with the commonly observed decreasing accuracy of the fold change values of the microarray method at the higher and lower ends. The correlation coefficients were 0.619 and 0.610 for the 200 ng and 500 ng samples, respectively. Red line represents the regression line.

## Discussion

In this study we evaluated the transcriptional consequences three weeks after a single neurotoxic dose of MDMA in DA rats with gene expression arrays. MDMA’s effects on the transcriptional level suggest alterations in cognition and memory related processes with the possible involvement of the CB1 and ephrin receptors in the HC. On the other hand, FC region exhibits more wide-scale changes in basic catabolic processes within FC cells and the upregulation of the 'dendrite development’ , 'regulation of synaptic plasticity’ and 'positive regulation of synapse assembly’ gene sets suggest a partial new synapse formation/synaptic reorganization in this region. These differences between the HC and FC indicate markedly different transcriptional responses of these two brain regions three weeks after a single dose MDMA administration.

### Hippocampus

In the HC we observed an upregulation of CB1 receptor mRNA. Nawata et al. also investigated CB1 receptor mRNA levels in the HC regions of mice up to 7 days following the cessation from repeated MDMA administration and they reported an increase 7 days, but not 1 day after the last treatment [43]. Our study shows that an increase of CB1 receptor levels can be caused even by a single-dose of MDMA and can be detected three weeks after the drug administration in rats. The presence of elevated CB1 receptor mRNA levels in both rats and mice, which have markedly different reactions to MDMA on the long-run [44], raises the possibility of such effects in human ecstasy users alike.

Selective serotonin reuptake inhibitor (SSRI) treatment is known to cause alterations in CB1 receptor levels in the HC [45,46] and these alterations might be the consequences of the altered serotonergic tone. Activation of serotonin 2C (5-HT 2C) receptors increases endocannabinoid production in the postsynaptic HC and amygdala neurons via the downstream activation of diacylglycerol (DAG) lipase [45]. The released 2-arachidonoil glycerol (2-AG) acts on the presynaptic neurons, and inhibits serotonin (5-HT) release through CB1 receptor activation thus forming a negative feedback loop [45]. MDMA treatment leads to a long-term serotonergic deficiency and to the damage of serotonergic axon terminals [2,5-7]. Hence, the result of the decreased endocannabinoid release from postsynaptic neurons might result in the observed upregulation of the CB1 receptor.

Cannabinoid agonists impair working memory and short term memory [36,39-41] and it has been also reported that MDMA can cause impairments in cognitive functions in humans, rats and mice [2,6,8-10,43]. Nawata et al. also showed that CB1 receptor antagonist attenuated the MDMA-induced cognitive deficit in mice [43]. Accordingly, we observed in the present study that genes involved in the regulation of memory and cognitive processes were downregulated after MDMA treatment in DA rats. The latter findings and the fact that both CB1 receptor elevations and cognitive deficits are present in multiple species suggest a central role of CB1 receptor and thus cannabinoid signaling in the reduced cognitive and memory functions following MDMA administration.

CB1 receptors exert their effects in the cells via calcium-signaling, thus upregulation of some of the calcium/calmodulin-dependent kinases (CAMK), calcium transporters, an inositol transporter and the phosphorylation gene set may be in association with CB1 receptor signaling. In addition, enhancement in cannabinoid signaling usually indirectly reduces glutamate release by acting on GABA-ergic interneurons in the HC (for a review see [47]). Accordingly, genes belonging to the regulation of the glutamatergic synaptic transmission were downregulated in the present study. Finally, elevated CB1 receptor signaling has been shown to impair neurite growth and arborization in developing rodent brain and cannabinoid agents in adult mice were able to modulate synaptic plasticity [48-50]. In accordance, we also observed downregulations in 'neuron projection development’ and synaptic plasticity related gene sets.

Here we also show upregulations of the mRNA levels of *Epha4*, *Epha5* and *Epha6* receptors in the HC after MDMA administration. These receptors have been reported to modulate synapse formation and glutamatergic long-term potentiation (LTP) (for a review see [51]). Since ephrin receptors are bidirectional receptors and regulate both presynaptic and postsynaptic neurons, the up- or downregulation of these receptors does not result in consequent elevation or suppression of synapse formation. Instead, a proper level of these receptors is required for accurate neuronal projection termination [52]. While *Epha4* and *Epha6* are widely expressed in the HC, *Epha5* is weakly labeled in this region under physiological conditions [53-55]. Epha4 was found to suppress synapse development in the HC [56], while *Epha5* knock-out (KO) mice showed decreased spine density in other brain regions [42] and may be necessary for proper hippocampal projections [57,58]. In another study, *Epha6* KO mice showed impaired cognitive functions [59]. Thus, it is clear that ephrin receptors modulate synapse formation in the HC and related cognitive functions.

### Frontal cortex

While alterations in the expression of 5-HT markers are well-defined, studies examining other effects of MDMA on gene expression are scarce. Thiriet et al. examined 1176, toxicology-related genes in adult Sprague–Dawley rats and followed expression patterns up to 7 days after a 20 mg/kg single-dose MDMA administration in the FC [60]. They found nerve growth factor alterations and suggested cytoskeletal reorganization while in another study by Fernandez-Castillo et al. emphasized neuroinflammatory responses in MDMA-effects 8 hours after repeated-administration in adult mice [61]. Martinez-Turillas et al. investigated brain-derived neurotrophic factor augmentations in the FC region of Wistar rats up to 7 days after drug administration [34]. In our present study we examined the gene expression patterns longer time (3 weeks) after a single neurotoxic dose of MDMA in the vulnerable DA rat strain. We report wide-scale downregulation of genes involved in chromatin organization, nucleocytoplasmic transport, ribosome-related functions, protein synthesis/folding and transmembrane transport processes in the FC region (Figure 5). It seems reasonable that the observed changes are the long-term consequence of the acute general neurotoxic processes, like toxic metabolite formation, hyperthermic effect or free radical production or the impairment in the autoregulation of cerebral blood flow [5,11-19]. The latter is even further supported by the upregulation of the response to hyperoxia gene set in the present study. We could not confirm neuroinflammatory changes [61] or BDNF dysregulation [34] observed by other authors in our experimental setup. In comparison with the previous study of Thiriet et al. [60], the growth factor activity gene set was upregulated, while some gene sets, related to neuronal cytoskeletal transport were downregulated in line with the previous study. However, this similarity existed only on the level of the mentioned biological processes, and was a result of the dysregulation of other genes, a possible result of the differences in the strain, time-scale and dosage regimen between the two studies.

Motor regions in the FC are targets of thalamical inputs and contribute to motor system functions [62]. Studies in DA rats with the same MDMA administration protocol like in the recent experiment indicated chronic changes in motor activity [63-65]. Additionally, Karageorgiou et al. reported alterations in right supplementary motor area activation in human MDMA users in an fMRI study [66]. These results might reflect subsequent impairments in motor functions on the long-run and are in accordance with the observed wide-scale changes in the recent experiment.

As from another functional perspective FC and prefrontal cortical regions (PFC) are not only responsible for motor functions, but are also closely related to different cognitive tasks, e.g. working memory, goal-directed behavior, and executive functioning in rats [26,67-69]. In our experiment FC samples contained regions from primary and secondary (supportive) motor cortices principally and likely some parts of the PFC [69]. Thus the inhibition of certain biosynthetic processes found in the present study may even participate in the cognitive decline of heavy MDMA users.

At the same time, however, upregulation of neurite formation related gene sets and thus a partial reinstatement of FC networks is also suggested by our present data. Additionally, the upregulation of HSP-related genes in the present study also suggests different extent in recovery processes. The latter results and the lack of similar processes in the HC might point out to different severity of damage of different memory types. Indeed, the only study investigating such differences following binge administration of MDMA, reported rats learning working-memory related tasks (mainly FC mediated) faster on the long-run compared to spatial reference memory (mainly HC mediated) in an 8-arm radial maze challenge [70].

Taken together, the downregulation of almost 50 gene sets related to biosynthetic processes in the FC may reflect transcriptional adaptations to well-known general neurotoxic effects not related to specific pathways 3 weeks after the drug administration. At the same time, the upregulation of the gene sets responsible for synapse/dendrite formation in this brain region may point to a starting new synapse formation/synaptic reorganization and might be a sign of a compensatory mechanism ameliorating MDMA’s acute effects 3 weeks after the administration.

### Dorsal raphe

The changes in the DR region were mild in line with our previous results suggesting that MDMA-caused damage to these neurons are restricted to serotonergic axon terminals instead of neuronal cell bodies directly [71]. The caspase activation gene set significantly changed in the present study was not supported by individual genes, or other gene sets related to apoptotical processes. The downregulation in 11beta-hydroxysteroid dehydrogenase type 1 mRNA levels might suggest a possible role of the hypothalamic-pituitary-adrenal axis in MDMA’s long-term consequences, an effect also proposed by others [72,73]. However, the DR region seems to be mostly unaffected 3 weeks after a single-dose of MDMA administration in DA rats.

### Limitations

In the present study we have not elucidated the temporal patterns of the mRNAs. Further studies are needed addressing the time course of the described alterations to elicit the causative relations of these transcriptional processes in details.

We could not confirm the decreased expression of serotonergic markers in the present study. Both 5-HTT and TPH mRNA levels were unaltered in the treatment group, which is in conflict with previous results: well established prolonged serotonergic depletion and decreased expression of serotonergic markers in both protein and mRNA levels after MDMA-treatment were demonstrated by our group earlier [5,6]. Here we can assume that the collection of DR samples was not precise enough and as we did not apply laser capture microdissection in this case, significant amount of surrounding tissue was perhaps cut out together with the DR and it may result a bias in the measurement of serotonergic markers. Notably, the decrease of 5-HTT expression, measured by quantitative in situ hybridization, was approximately -20% in the same animal model 3 weeks after the MDMA treatment, compared to the control level, and this moderate alteration was significant only in case of the fine measurement of grain densities of individual cells but not with the measuring of the autoradiography signal on film [6].

On the other hand, microarray method has well-known drawbacks, when compared to polymerase chain reaction methods or immunohistochemistry used in our earlier papers. Namely, the limited amount of probes on the microarray may result in smaller fold change values, when compared to polymerase chain reaction methods (PCR), which can also be noticed on Figure 7. On the other hand, the shorter oligomers used can result in more mismatch hybridization, which can overcome smaller changes in gene expressions, like that in the case of 5-HTT. However, for this very reason we assume that the results presented here, with our strict significance criterion, are robust enough to overcome this bias.

**Figure 7:** **Correlation between the microarray and the Fluidigm GEx PCR array data.** The figure summarizes the correlation between the logarithmic microarray data and the validation results for both the 200 ng and 500 ng samples. For validation purposes we used the polymerase chain reaction-based (PCR-based) Fluidigm GEx array with 19 genes and upon receiving the results, the numerical analysis was performed with the inbuilt corr.test function of the R statistical computing program. The results are in agreement with the commonly observed decreasing accuracy of the fold change values of the microarray method at the higher and lower ends. The correlation coefficients were 0.619 and 0.610 for the 200 ng and 500 ng samples, respectively. Red line represents the regression line.

We did not find alterations in the BDNF gene expression, which is in agreement with our previous study where we demonstrated that (after a slight transient acute decrease) BDNF protein level was increased only 8 weeks after the same MDMA dosage regimen in the same rat strain [35].

We must also note the major limitation of transcriptomic studies, namely, mRNA levels do not necessarily reflect for the appropriate protein levels.

## Conclusion

We performed a genome-wide evaluation of transcriptional changes 3 weeks after a single-dose of MDMA in DA rats. Our results highlight CB1 and ephrin receptors as potential downstream mediators of MDMA in the HC. In addition, GSEA showed downregulation of the ‘cognition’ and ‘memory’ gene sets and also indicated a decreased functionality of long-term potentiation and the possible involvement of the hippocampal glutamatergic pathway in these processes. However, determination of causative relations or possible interactions between the observed changes requires further investigations.

On the other hand, the FC region showed markedly different changes. The differences compared to the HC were obvious by both the GSEA and by the heatmap analysis. These differences may reflect for the different anatomical properties/connectivity and also the different neurotransmitter contents of these regions. The downregulated pathways in the FC were related to the basic mechanisms of the cell functionality in the absence of specific markers of certain pathways. In the FC the upregulation of the ‘dendrite development’, ‘regulation of synaptic plasticity’ and ‘positive regulation of synapse assembly’ gene sets raise the possibility of new synapse formation/synaptic reorganization mechanisms in this region. In contrast, these gene sets were not upregulated in the HC. All of these results point out to a starting reinstatement of the neuronal pathways and connections in the FC, but not in the HC, three weeks after a 15 mg/kg dose of MDMA.

## Methods

### Animals

The animal experiments and housing conditions were carried out in accordance with the European Community Council Directive of 24 November 1986 (86/609/EEC), as well as the National Institutes of Health Principles of Laboratory Animal Care (NIH Publication 85–23, revised 1985) and special national laws (the Hungarian Governmental Regulation on animal studies, 31 December 1998 Act). The experiments were approved by the National Scientific Ethical Committee on Animal Experimentation and permitted by the Food Chain Safety and Animal Health Directorate of the Central Agricultural Office, Hungary (permission number: 22.1/3152/001/2007).

Altogether 21 male DA rats (Harlan, Olac Ltd, Shaw’s Farm, Blackthorn, Bicester, Oxon, UK) aged approximately 8 weeks (weighing 152 ± 3,58 g (SEM) at the beginning of the experiment) were used. The animals (four per cage) were kept under controlled environmental conditions along the whole experiment (temperature 21 ± 1°C, humidity: 40-50%, 12 hour light–dark cycle starting at 6:00 a.m.) and food and water were available for them ad libitum.

### Drug administration and experimental design

(±)3,4-methylenedioxymethamphetamine (Sanofi-Synthelabo-Chinoin, Hungary, purity >99.5%) was dissolved in 0.9% NaCl (SAL) at an equivalent dose of 15 mg/kg free base and was administered intraperitoneally (i.p.) in a volume of 1 ml/kg. For control animals SAL was used i.p. in equivalent volumes (1 ml/kg).

The MDMA-treated and control groups consisted of 11 and 10 animals, respectively, and were randomly assigned to each group. Vehicle-containing Alzet 2001 osmotic minipumps (Durect Corp., CA, USA) were inserted under the skin for all animals. The rats were sacrificed 3 weeks after the injections.

### RNA extraction and sample preparation

Three weeks after MDMA or vehicle injections rats were killed quickly by decapitation. The brains were removed, approximately 2 mm thick coronal sections were cut and the HC, FC and DR regions were dissected according to Paxinos and Watson ( [74], dorsal HC: from bregma -2.5 mm to -4.5 mm; FC: from bregma +1.7 to -0.3 mm; DR: from bregma -7 mm to -8 mm, respectively) and stored at -80°C. The samples were homogenized with 1 ml TRIzol reagent (Ambion, TX, USA) according to the manufacturer’s instructions. Thus, the homogenized samples were centrifuged at 12000 g at 4°C for 10 minutes, the supernatant transferred to a new sterile Eppendorf tube and incubated at room temperature for 5 minutes. Chloroform in a volume of 200 μl was added; the mixture was vortexed and incubated again at room temperature for 2–3 minutes. Following centrifugation at 12000 x g at 4°C for 15 minutes the upper (clear) aqueous phase was transferred to a new Eppendorf tube and was mixed with 500 μl of isopropranol and incubated for 10 minutes at room temperature. After centrifuging the samples at 12000 x g at 4°C for 10 minutes the supernatant was removed and 1 ml 75% ethanol was added to the precipitation. The samples were again centrifuged at 7500 x g at 4°C for 5 minutes, the supernatant was removed, and 1 ml 75% ethanol was added. After centrifuging samples at 7500 x g at 4°C for 5 minutes, the ethanol was removed, and the RNA pellets briefly dried. The pellets were dissolved in 20 μl diethylpyrocarbonate treated-dH_2_O (DEPC-dH_2_O) and the samples stored at -80°C until further processing.

To determine the quality of the samples 1–2 μl were used for optical density (OD, 260/230 and 260/280 ratios) measurements. The OD ratios were determined for all samples and randomly repeated to evaluate the reliability of the measurements (no significant difference was observed, data not shown). Samples with the lowest RNA concentrations were excluded from further analysis and thus both MDMA and control groups consisted of 8 animals. Two-two randomly selected samples were pooled in each treatment group resulting in 4 pooled samples per brain region and per treatment group. These samples (altogether 24 samples) were sent to Service XS (Leiden, Netherlands) for microarray analysis with the Illumina (San Diego, CA, USA) RatRef-12 v1 beadarray expression chip. Upon arrival, samples were once again subjects to a purification process and quality control measurements with Agilent Bioanalyzer and Nanodrop spectrophotometer and one sample from the DR region was excluded from further analysis due to degradation.

### Data analysis

Raw microarray data were processed with beadarray [75], preprocessCore [76] and puma [77] Bioconductor [78] packages for R [79] as described in [80]. Briefly, backgroundCorrect method used in the beadarray package was set to "minimum", and "log = TRUE; n = 10" variables were used for createbeadsummaryData method. The normalization method used was the quantile normalization method in the preprocessCore package. Additionally, pumaComb, pumaDE, and write.rslts functions with default settings were used. Changes were considered statistically significant when the MinPplr was below 0.001. This strict criterion was necessary to reduce the number of false positive results to an acceptable limit.

Heatmap visualization of the differences in gene expression was done using Multiexperiment Viewer Tool [81,82]. Genes with similar expression patterns are grouped together with hierarchical clustering (Euclidean distance, average linkage) [83].

GSEA was performed using GSEA version 3.1 from the Broad Institute at MIT ( http://www.broadinstitute.org/gsea) [84,85]. Gene sets (GMT format) were obtained from the MSigDB for C5 category (GO gene sets) and in addition, neuronal function related gene sets were selected from the GO homepage ( http://www.geneontology.org; [86]) manually. Gene identifiers used in the array dataset and gene sets were gene symbols. The data set had 22523 features (Illumina probes), which were collapsed to gene symbols (the median expression value was used for the probe set). In these analyses, the gene sets analyzed were restricted to those sets containing between 15 and 500 genes as recommended [87]. The t-test was used as the metrics for ranking genes and gene set was chosen as the permutation type since the sample size was less than 7 in this study. 1000 permutations were used to calculate p-value with the seed of permutation set to 149. All other basic and advanced fields were set to default.

A normalized enrichment score (NES) was calculated for each gene set to represent the degree in which it was enriched in one phenotype. The nominal p-value and the FDR corresponding to each NES were calculated. A NES with a nominal p-value <0.05, FDR <0.25 were considered statistically significant.

Network visualization and analysis using enrichment results was done using Cytoscape 2.8.3. and its plugin "Enrichment Analyzer" with the following cut-offs: similarity coefficient cut-off 0.1, p-value cut-off 0.05 and FDR cut-off 0.25 [88,89].

### PCR validation

We have validated altogether 19 RNA products from the original pooled samples with real-time PCR on Fluidigm GEx array (San Francisco, CA, USA) using Taqman Gene Expression assays for the appropriate RNAs obtained from Applied Biosystems (Carlsbad, CA, USA) (for the full list of validated genes see Additional file 4: Table S4). Each sample was used in duplo following quality control measurements (altogether three samples were excluded due to degraded or insufficient amount of RNA). The validation experiment was performed by Service XS (Leiden, Netherlands). Upon arrival of the normalized results, manually written R scripts using the cor.test function with default settings were used for the comparison between microarray and PCR data. The Pearson correlation coefficients were 0.619 and 0.610 for the 200 ng and 500 ng samples, respectively. In both cases p-values were far below 0.001. The linear regression is depicted on Figure 7.

### Availability of supporting data

The data supporting the results of this publication have been deposited in NCBI’s Gene Expression Omnibus [90] and are accessible through GEO Series accession number GSE47541 ( http://www.ncbi.nlm.nih.gov/geo/query/acc.cgi?acc=GSE47541).

## Abbreviations

2-AG: 2-arachidonoylglycerol; 5-HT: Serotonin; 5-HT 2C: Serotonin 2C receptor; 5-HTT: Serotonin transporter; CAMK: Calcium/calmodulin dependent kinases; CNS: Central nervous system; CB1: Cannabinoid receptor type 1; DA: Dark Agouti; DAG: Diacylglycerol; DEPC: Diethylpyrocarbonate; DR: Dorsal raphe; FC: Frontal cortex; FDR: False discovery rate; GEO: Gene Expression Omnibus; GO: Gene ontology; GSEA: Gene set enrichment; HC: Hippocampus; HSPs: Heat-shock proteins; i.p.: Intraperitoneal; KO: Knock-out; LTP: Long-term potentiation; MDMA: 3,4-methylenedioxymethamphetamine; MinPplr: Minimum probability of positive log ratio; NES: Normalized enrichment score; nomP: Nominal p-value; OD: Optical density; PCR: Polymerase chain reaction; PFC: Prefrontal cortex; SAL: Saline; SEM: Standard error of the mean; SSRI: Selective serotonin reuptake inhibitor; TPH: Tryptophan hydroxylase; TRP: Transport (in figures); TRPER: Transporter (in figures).

## Competing interests

The authors declare that they have no competing interests.

## Authors’ contributions

PP participated in the GSEA analysis and organized the PCR validation, wrote the R scripts, interpreted the data and drafted the manuscript. VT carried out the GSEA analysis and participated in the interpretation while also contributed in drafting of the manuscript. CA, EK, RDA carried out the treatment protocol dissected the brain samples and prepared the RNA extractions. LT helped in data analysis, to draft the manuscript and contributed to the written R scripts. GB prepared the study design and protocols, coordinated the study and helped in the interpretation and drafting of the manuscript. All authors have read and approved the final manuscript.

## Supplementary Material

Additional file 1: Table S1 Contains significantly up- or downregulated genes compared to the control group in the three examined brain region. Click here for file

Additional file 2: Table S2 Contains individually selected GO terms for GSEA analysis. Click here for file

Additional file 3: Table S3 Contains the significantly enriched GO terms selected by NES, FDR and nominal p-values (nomP) in the examined brain regions. Click here for file

Additional file 4: Table S4 Contains the genes validated with the Fluidigm GEx PCR array and the used TaqMan assays. Click here for file
